# Based on Contaminated Water and Human Health to Change of China's International Image Under Mainstream Media Reports During the COVID-19 Pandemic

**DOI:** 10.1155/2022/7537056

**Published:** 2022-08-23

**Authors:** Kaixi Ji, Mengqian Zhou, Zitong Yang, Haiyong Zong

**Affiliations:** ^1^School of Liberal Arts, Nantong University, Nantong 226000, China; ^2^School of Marxism, Nantong University, Nantong 226000, China

## Abstract

As water quality can be an indicator of public health, it cannot be ignored. We can regard the international image of a country as a kind of soft national power, which embodies the comprehensive strength of the country and plays a very important role in safeguarding the interests of a country. This article aims to study the changes in China's international image under mainstream media reports during the COVID-19 pandemic. This article is based on contaminated water and human health to study the concept of the international image, the optimization path of China's international image, and the SEIR model. The SEIR model is one of the classic infectious disease models. Because the virus infection rate in this model is constant, it is difficult to accurately determine the spread of new coronary pneumonia. To model and complete the pandemic trend prediction and other issues, this article proposes a virus infection rate prediction method based on the long short-term memory network (LSTM), and combines it with the SEIR model to establish a new crown pneumonia pandemic trend prediction model (LS-Net). The conclusion of this article shows that in the fight against the novel coronavirus infectious pneumonia pandemic, the Chinese people have demonstrated the style of a big country. I have unreservedly passed on my own experience in pandemic prevention and control to countries around the world, and dispatched medical teams to provide the world with Chinese “prescriptions.” Chinese diagnosis and treatment programs are the crystallization of common wisdom of Chinese medicine and Western medicine to support the world. All countries fight the pandemic together. In this analysis, Pakistan, Kenya, and Nigeria hold 84%, 85%, and 75% of China's positive views, respectively, 61% of Russians also have a positive attitude toward China.

## 1. Introduction

### 1.1. Background of Topic Selection

As China has made a huge contribution to the world's new crown pandemic, mainstream media's attention to China has gradually increased, reports have continued to increase, and the scope of coverage has continued to expand. In particular, the rapid rise of mainstream media reports during the COVID-19 pandemic has given coverage and content. Both methods have undergone profound changes. China's internal affairs and diplomatic performance have been well received by mainstream media during the COVID-19 pandemic. China's international influence has gained wider attention and recognition. A comprehensive, objective, and true image of modern China is being formed during the COVID-19 pandemic. The development of the media is becoming more and more diversified. All of this makes the sense of time and space between countries, between countries and citizens, and social organizations so weakened.

### 1.2. Significance of the Research

The research significance of this article is to classify and analyze the current research on the construction of China's international image under mainstream media coverage during the new crown pandemic from a micro and macro perspective, and to conduct a more systematic and in-depth study of this topic. The previous research is needed to put forward its point of view to supplement the current gaps in related research. The main body of this research is the media. It not only includes the analysis of cases of international media communication behaviors, but also systematically studies the communication of national image building with the participation of the database, and studies the international media communication. On this basis, I would like to supplement the research on the “national image” from the perspective of news and communication to the relevant analysis of the Chinese media in shaping and enhancing China's national image, and hope to use this as a basis. Put forward overall directions for future in-depth research.

### 1.3. Work Related to the Changes in China's International Image

In the fight against the novel coronavirus infectious pneumonia pandemic, the Chinese people have demonstrated the style of a big country. Unreservedly spread their own experience in pandemic prevention and control to countries around the world, dispatched medical teams to support countries around the world to jointly fight the pandemic, and provide the world with China's “prescription” Chinese diagnosis and treatment plan is a joint fight against the pandemic by Chinese and Western medicines. Hartig studies the hegemonic narrative advocated by the mainstream media, the content is China's response to the COVID-19 pandemic and its facts. The COVID-19 pandemic has triggered multidimensional crises including public health and political economy. Disagreements between countries on public health and economic policy responses have led to a propaganda war. After roughly examining the time trajectory of China's public health response and its underlying factors, this article continues to study some controversial issues regarding China's public health response to the COVID-19 pandemic highlighted in hegemony [1]. However, our understanding of the dynamics of this exposure response during the COVID-19 pandemic is still limited. Benabdallah believes that the elderly have received great media attention during the COVID-19 pandemic because they are considered susceptible to this new virus based on clinical data and epidemiological evidence. A large number of media reports have played an important role in calling for the improvement of public health services for the elderly population. However, during a pandemic, problematic media coverage of the elderly may cause or exacerbate age discrimination. Therefore, this study uses empirical data collected from five mainstream media in China from January 3 to May 3, 2020, to study how the media constructs the vulnerability of the elderly and their potential age perception during the pandemic. The survey results show that the media clearly tends to portray the elderly as passive recipients, while seeking resources from families, public institutions, and governments at all levels to deal with the COVID-19 pandemic [2]. Niu researches that the exposure and consumption of information during an pandemic may change perceptions of risk, trigger changes in behavior, and ultimately affect the development of the disease. Therefore, it is very important to disseminate map information through mainstream media and public response [3]. However, our understanding of the dynamics of this exposure response during the COVID-19 pandemic is still limited.

### 1.4. Innovation Points of This Research

1. China's international image has undergone tremendous changes under mainstream media reports during the COVID-19 pandemic. In the fight against the novel coronavirus-infected pneumonia pandemic, the Chinese people have demonstrated the style of a big country. Unreservedly spread their own experience in pandemic prevention and control to countries around the world, dispatched medical teams to support countries around the world to jointly fight the pandemic, and provide the world with China's “prescription” Chinese diagnosis and treatment plan is a joint fight against the pandemic by Chinese and Western medicines. The crystallization of common wisdom makes people all over the world look at the Chinese with admiration.
2. The SEIR model is one of the classic infectious disease models. Because the virus infection rate in this model is constant, it is difficult to accurately model the spread of new coronary pneumonia and complete the pandemic trend prediction. In response to this problem, this article proposes a virus infection rate prediction method based on long short-term memory (LSTM) network, and combines it with the SEIR model to establish a new crown pneumonia pandemic trend prediction model (LS-Net).

## 2. Method of the Change of China's International Image

### 2.1. Concept of International Image

The research on international image mainly focuses on the external construction of the country itself [4]. External construction includes international self-construction and feedback from the international media on the international image. The main audience of the international image includes not only the nationals of the country, but also the international exchanges abroad. China's media and national image have different forms in different media [5]. The representative views of foreign scholars on the definition of the national image are mainly shown in Table 1.

It can be seen that the concept of international image is an open and variable concept, and different scholars have different definitions of it in different periods. According to the definition of the above scholars, the author believes that the international image is the result of the combination of “self-shaping” and “other shaping.” It is dynamic, including images at home and abroad, with different cognitive themes, cultural backgrounds, and values and information. Depending on the channel, the domestic image and the foreign image are usually different [6].

### 2.2. Role of International Image

The international image is the embodiment of a country's comprehensive national strength. In today's world of economic globalization and political diversification, shaping and maintaining a good international image is the expectation of every country. International image is the passport of a country entering the international arena. The role of enhancing the internal demand of the country's overall national strength and international image can be explained from the following two perspectives:

1. Economically, with the development of economic globalization, trade cooperation and competition between countries have become the norm [7]. In recent years, China's position in the international economy and trade has become more and more important, especially with the launch of the Asian Investment Bank and the “One Belt, One Road” strategy proposed by China this year [8]. A good country image helps promote trade between the country and other countries.
2. From a social and cultural perspective, a good national image can create a positive, friendly, peaceful, and profitable atmosphere, and play an important role in the development of a country's culture [9]. In recent years, the rise of Chinese, the increase in the number of Chinese students studying abroad, and the establishment of Confucius Institutes around the world may all reflect the influence of China's national image on promoting social and cultural exchanges between the two countries.

### 2.3. Optimization Path of China's International Image

General Secretary Xi Jinping once pointed out that “it is necessary to promote the construction of international communication capacity, tell Chinese stories, spread Chinese voice, show the world a true, three-dimensional and comprehensive China, and improve the country's cultural soft power and Chinese cultural influence [10].” West The image of society's prejudice against China has not been eliminated with the rise of China's economy. China's national image is still largely shaped by Western media, even though China has tried to change this through a series of official and private measures. With the global outbreak of the new crown pneumonia pandemic, Western public opinion is still full of prejudice, discrimination, and ideological struggles in shaping China's image. Therefore, China needs to change this phenomenon by optimizing the international image shaping path, as shown in Figure 1.

#### 2.3.1. Improve the Level of Domestic Crisis Handling

Whether it was the SARS pandemic in 2002 or the new crown pneumonia pandemic, there were problems that local governments did not handle well at the beginning of the pandemic. Mistakes in the work of local governments caused the masses to lose confidence in the openness and transparency of government information. Negative public opinion is often adopted by Western media and continuously amplified, which ultimately leads to the deterioration of China's international image [11]. Therefore, in shaping China's excellent image internationally, the most important thing is to continuously improve the level of domestic local governments in dealing with major crises, and to guide rational public opinion through the effective implementation of General Secretary Xi Jinping's people-centered thinking. Solve the problem of external factors through continuous improvement of internal factors [12].

#### 2.3.2. Flexible Application of Social Media Platforms

In the era of the popularization of smartphones, social media platforms have become one of the main sources for ordinary people to obtain information, and social media is the only way for a very large number of young people. Due to low cost and high speed, social media platforms have become the main channel for the spread of major emergencies [13]. Due to the different ways of information publishing and dissemination subjects, information on social media platforms is mixed, and many messages are full of prejudice and discrimination. Relevant departments of the Chinese government should flexibly use various social media platforms to publish relevant news instantly and transparently, leading the trend of public opinion and avoiding similar incidents like Dr. Li Wenliang [14].

#### 2.3.3. Properly Handle False News Immediately

In the context of the Internet age, the West will pay attention to false news in China and expand it through social media platforms and other channels, which will eventually lead to prejudice, discrimination, and racism [15]. Relevant departments of the Chinese government should respond to all kinds of false news in a timely manner, by inviting domestic and foreign experts in relevant fields and dealing with all kinds of false news, through scientific research and judgment, clarifying to the people at home and abroad, combining with the use of social media platforms. The false remarks of the Western media counterattacked, destroying the West's intention to discredit China's image [14].

#### 2.3.4. Change the International Image Publicity Strategy

In the past, China mainly used the dissemination of historical culture and natural scenery to shape China's international image, rather than contemporary China's development stories. In the context of the new crown pneumonia pandemic, China's political system has frequently become the target of Western media attacks. Therefore, China is bound to strengthen the advantages of the system and establish an international image communication strategy with contemporary China as the main body [16]. The masses should be guided and encouraged to publicize the advantages of China's system on various Internet media, to form China's international Internet voice, and to refute the false statements of the West that slander China's image. By telling the story of contemporary China, it shows China's contribution to the fight against the new crown pneumonia pandemic and other major international events, and constantly uses vivid deeds to shape China's responsible international image and spread the concept of a community with a shared future for mankind [17].

### 2.4. Infectious Disease Transmission Model: SEIR

The SEIR model is a classic infectious disease model. It divides the population into four categories: infected (I), the total number of confirmed patients who have been infected with the virus and have symptoms; removed (R), the total number of people who die or are successfully cured after being infected with the virus; susceptible (S), the total number of healthy people who may be infected with the virus; and exposed (E), the total number of people who have been infected with the virus but still have no symptoms. In the COVID-19 pandemic, the transformation relationship of the four groups of people in the SEIR model is shown in Figure 2. In the figure, *β*_1_ is the probability of the latent person transmitting the virus to the susceptible person and *β*_2_ is the probability of the infected person transmitting the virus to the susceptible person, *α* is the probability of a latent person being transformed into an infected person, and *γ* is the probability of an infected person being transformed into a remover. The kinetic equation of SEIR is:

(1) $$\begin{array}{c} \frac{\text{d}S}{\text{d}t}=-\frac{-b_{1}SE}{N}-\frac{-b_{2}SI}{N}, \end{array}$$

(2) $$\begin{array}{c} \frac{\text{d}E}{\text{d}t}=\frac{b_{1}SE}{N}+\frac{b_{2}SI}{N}-aE, \end{array}$$

(3) $$\begin{array}{c} \frac{\text{d}I}{\text{d}t}=aE-gI, \end{array}$$

(4) $$\begin{array}{c} \frac{\text{d}R}{\text{d}t}=gI. \end{array}$$

In the equation, *t* is the time step; *N*=*S* + *E* + *I* + *R*, which is the total number of people.

The calculation method of virus infection rate *β*_1_, *β*_2_ is calculated by equation (5):

(5) $$\begin{array}{c} \beta_{1}=k_{1}b,\\ \beta_{2}=k_{2}b. \end{array}$$

In the formula, *k*_1_ and *k*_2_ are the average number of people in contact with each latent person and each infected person each day; *b* is the transmission rate of the virus, which can be calculated by the SIR model. The SIR model is similar to the SEIR model. It divides the population into three categories: susceptible, infected, and removed. In the SIR model, since the number of people infected is small at the beginning of the virus infection, *N* is approximately equal to *S*:

(6) $$\begin{array}{c} \frac{\text{d}I}{\text{d}t}=\frac{\beta SI}{N}-\gamma I\approx \left(\beta -\gamma \right)I. \end{array}$$

From formula (6), we can get:

(7) $$\begin{array}{c} I\left(t\right)=\exp\left[\left(kb-\gamma \right)I\right]. \end{array}$$

From equation (7), *b* can be calculated, and by putting it into equation (5), *β*_1_ and *β*_2_ in the SEIR model can be calculated.

In the traditional SEIR model, *β*_1_ and *β*_2_ are often constants derived from data statistics. In reality, the infectious ability of the virus will be greatly affected by the outside world, so *β*_1_ and *β*_2_ should be constantly changing [18]. In the above method, both *β*_1_ and *β*_2_ are calculated by the SIR model, and the virus infection of patients during the incubation period is not considered.

### 2.5. New Crown Pneumonia Pandemic Trend Prediction Model: LS-Net

Aiming at the problem that the virus infection rate in the traditional SEIR model cannot be automatically and dynamically predicted and the infection status of patients in the incubation period is not considered, this article proposes LS-Net [19, 20] based on the LSTM and SEIR models. This section will introduce LS-Net in detail.

The overall structure of LS-Net is shown in Figure 3. It contains two modules: a virus infection rate prediction module and an pandemic trend prediction module. The pandemic trend prediction module includes the SEIR model layer to realize the prediction of the new crown pandemic trend [21]. The virus infection rate prediction module includes an LSTM layer, a fully connection (FC) layer, and a nonlinear transformation layer to realize the prediction of the new coronavirus infection rate *β*_1_ and*β*_2_.

The virus infection rate prediction module is based on LSTM and predicts the infection rate based on the law of virus transmission. In order to better learn the correlation information between time series data, LS-Net uses the three-day incubation period, the number of infected persons, and the number of removed persons as input. The later changes of the virus infection rate are closely related to the prevention, control, diagnosis, and treatment measures in the early stage of the pandemic. Therefore, the prediction of the virus infection rate needs to be combined with historical information and current information to be analyzed together [22, 23]. LSTM can learn and generate data containing historical information and current information. It includes three types of gates: input gate *i*_*t*_, forget gate *f*_*t*_, and output gate *o*_*t*_. The LSTM update process is shown in equations (8)–(13), *X*_*t*_ is the input at time *t* [24].

(8) $$\begin{array}{c} i_{t}=s\left(W_{ii}X_{t}+b_{ii}+W_{hi}h_{i-1}+b_{hi}\right), \end{array}$$

(9) $$\begin{array}{c} f_{t}=s\left(W_{if}X_{t}+b_{if}+W_{hf}h_{i-1}+b_{hf}\right), \end{array}$$

(10) $$\begin{array}{c} {\tilde{c}}_{t}=s\left(W_{ii}X_{t}+b_{i\tilde{c}}+W_{hi}h_{i-1}+b_{h\tilde{c}}\right), \end{array}$$

(11) $$\begin{array}{c} o_{t}=s\left(W_{io}X_{t}+b_{io}+W_{ho}h_{i-1}+b_{ho}\right), \end{array}$$

(12) $$\begin{array}{c} c_{t}=f_{t}c_{t-1}+i_{t}{\tilde{c}}_{t}, \end{array}$$

(13) $$\begin{array}{c} h_{t}=o_{t}\tanh\left(c_{t}\right). \end{array}$$

Input the features containing timing information output by *h*_*t*_ into the FC layer. The FC layer calculation process is shown in equation (14), where *C*_*t*_, *a*_*t*_, and *k*_*t*_ are all control parameters for predicting *β*_1_ and *β*_2_ at time *t*.

(14) $$\begin{array}{c} \left\{\begin{array}{c} C_{t}=\mathrm{lg}\left(1+\exp\left(W_{C}h_{t}\right)\right)\\ a_{t}=\mathrm{lg}\left(1+\exp\left(W_{a}h_{t}\right)\right)\\ k_{t}=\mathrm{lg}\left(1+\exp\left(W_{k}h_{t}\right)\right) \end{array}\right). \end{array}$$

## 3. Experiments on the Response of the Chinese People during the New Crown Pandemic

### 3.1. Research Experiments in the Context of the New Crown Pandemic

In December 2019, new coronary pneumonia (COVID-19) was successively discovered in Hubei Province and other parts of the country. With further development over time, the number of confirmed and suspected patients has continued to increase. After the outbreak of the new crown pneumonia pandemic, the impact of pandemic has brought an impact on the public's psychology. The new coronary pneumonia has become a public health emergency of international concern. The National Health Commission issued Announcement No. 1 on January 20, 2020, including pneumonia caused by the new coronavirus into the Class B infection stipulated in the “Law of the People's Republic of China on the Prevention and Control of Infectious Diseases.” However, the prevention and control measures of Class A infectious diseases shall be adopted, and they shall be included in the management of quarantine infectious diseases. After the outbreak of the new crown pneumonia pandemic, the impact of the pandemic has brought an impact on the public's psychology. The outbreak of the new crown pneumonia caused the entire China to press the pause button, and more than one billion Chinese people were trapped at home. Everyone controls not to go out. You must also wear a mask when you go out, so as to prevent yourself from being infected and to reduce trouble for the country. The new coronary pneumonia picture is shown in Figure 4.

### 3.2. Differences in Mental Health Among People in Different Regions Under the Pneumonia Pandemic

Using a factor of variance to analyze different aspects of the mental health of people outside Hubei Province, Wuhan City, it shows that people in different regions have no significant differences in the degree of fear and the level of stress. There is no significant difference in the degree of anger among people in the region. However, there are significant differences in the degree of depression among people in different regions. Further comparative analysis after multiples found that there are significant differences in the size of individual depression in areas outside Hubei and Wuhan, as shown in Table 2.

The independent sample *t*-test was used to further analyze the differences in the various dimensions of mental health among people of different genders in different regions. The results show that there are significant differences in the fear and anxiety dimensions of the mental health scale for individuals of different genders in Wuhan, and women have higher levels of fear and anxiety than men. Individuals of different genders in Hubei non-Wuhan area only have significant differences in the dimension of fear, among which the fear level of women is significantly higher than that of men. Individuals of different genders outside Hubei have significant differences in the dimensions of fear, anxiety, and anger. Among them, the level of fear, anxiety, and anger of women is significantly higher than that of men as shown in Table 3.

### 3.3. Differences in Mental Health among People of Different Occupations Under the Pneumonia Pandemic

An independent sample *t*-test was used to analyze the different dimensions of the mental health of people in different occupations. It shows that people of different occupations have no significant differences in the dimension of fear and depression, and people of different occupations are in the dimension of anxiety. The difference is not significant; people of different occupations do not have significant differences in the dimension of anger as shown in Table 4.

### 3.4. Differences in Mental Health Among People of Different Ages Under the Pneumonia Pandemic

Using one-way variance to analyze the different dimensions of people's mental health at different ages shows that there is no significant difference in the dimensions of fear, depression, anxiety, and anger as shown in Table 5.

## 4. Changes in China's International Image

### 4.1. Situation Under Mainstream Media Reports at the Beginning of the Outbreak of the New Crown Pneumonia

In the early stage of the outbreak of the new crown pneumonia pandemic, the mainstream media in the West mostly reported negative images of China. They can be divided into three categories. The first category is “regionalization,” which links the virus with China to make ordinary people feel more about China. Views are “viralized.” The second type is “politicization,” which is to combine the spread of the pandemic with China's political system to attack China's political system. The third type is “failed,” that is, to criticize China's adoption of the double standards act and turn a blind eye to the success achieved. Through three methods of reporting, Western media has portrayed China as an “undemocratic and irresponsible dictatorship” country, which is widely disseminated among ordinary people.

### 4.2. China's International Image After the Successful Control of the New Crown Pneumonia Pandemic

After the new crown pneumonia pandemic has spread globally on a large scale, the domestic situation in China is in sharp contrast with that in Western countries. Against this background, there have been fewer and fewer reports of demonizing and stigmatizing China's image in the early stages of the outbreak of the new crown pneumonia pandemic, and China's international image has gradually become a “leadership role” in the reports of mainstream Western media as “Great country.” The number of new cases in China has been declining, and the number of cases in most provinces has been cleared. The prevention and control of the new crown pneumonia pandemic have achieved initial success. However, because Western countries have not taken decisive and resolute actions, the number of new cases has continued to rise in the hardest hit area of the pandemic.

### 4.3. China's International Image Before and After the Pandemic

According to surveys conducted in 22 countries/regions (excluding China), more and more people in 15 of 21 countries believe that China is positive. China has a better image among the people of the Arab world, Africa, Latin America, and other developing countries, especially Pakistan, Kenya, and Nigeria. About 84%, 85%, and 75% of these three countries are optimistic about China and 61% of Russians also have a positive attitude toward China. Among Western countries, Americans believe that China is the most active country, accounting for 48%. Spain and the United Kingdom are slightly lower, but generally positive. More people in France, Germany, and Japan hold negative views of China than those who hold positive views. The most important reason for China to maintain an overall positive international image is that China's economy continues to grow rapidly, followed by many events, such as the Beijing Olympics and the Shanghai World Expo. More and more people come and visit China and learn about China. In addition, it is China that is gradually assuming more international responsibilities and is committed to solving international problems. This is why China has a better image. The details are shown in Figure 5.

### 4.4. Overseas Spread of the New Crown Pneumonia Pandemic

The new coronary pneumonia pandemic has been brought under control in China, but its spread abroad is accelerating, and Europe has become a “severe disaster area.” After the World Health Organization (WHO) announced the new pneumonia pandemic as “PHEIC” on January 30, local time, on March 12, the WHO further announced that the new coronary heart disease pandemic had become a “global pandemic.” According to data from the World Health Organization, as of March 19, the new rosette pandemic has spread to more than 150 countries or regions, with a total of 209,839 confirmed cases worldwide, and the number of new confirmed cases outside China far exceeds that in China, 16,498. The situation of pandemic prevention and control abroad is unacceptable. Among them, there are more than 1,000 people infected with the virus in 15 overseas countries. Italy has become the country with the worst pandemic abroad, with 35,713 confirmed cases. Other countries such as Iran, Spain, South Korea, France, Germany, and the United States are also accelerating. The comparison of the number of new cases per day between China and outside China is shown in Figure 6.

### 4.5. Impact of the New Crown Pneumonia Pandemic on the World Economy

The impact of the pandemic on macroeconomics is mainly reflected in two aspects: first, the spread of panic has led to a reversal of investor confidence, which has disturbed the financial and capital markets; second, the control of quarantine measures has put pressure on the macro economy. Therefore, pressure is exerted on both the consumer and the producer. We will analyze the impact of the pandemic from the spread of the pandemic in the capital market, trade, industrial chain, and cross-border investment. The schematic diagram is shown in Figure 7.

## 5. Conclusion

In the fight against the novel coronavirus infectious pneumonia pandemic, the Chinese people have demonstrated the style of a big country. First, I have unreservedly passed on my own experience in pandemic prevention and control to all countries in the world, and at the same time, I have unreservedly dedicated my treatment experience to all countries in the world. Second, when the pandemic situation in other countries was severe and medical resources were in short supply, the country dispatched medical teams on time to support countries around the world to fight the pandemic together. Therefore, China has made a selfless dedication to all countries in the world in the fight against the novel coronavirus pneumonia pandemic. Third, provided the world with China's “prescription,” Chinese diagnosis and treatment programs are the crystallization of common wisdom and common wisdom between Chinese and Western medicine to fight the pandemic together. In the treatment plan, Chinese medicine has a relatively important position. Traditional Chinese medicine has unique theories and practices in preventing and treating the plague. It is an effective treatment method to give full play to the overall regulation of traditional Chinese medicine, improve immunity, and stimulate one's own disease resistance and rehabilitation capabilities. Fourth, the World Health Organization believes that China has adopted the bravest, most flexible, and most active prevention and control measures in history, which has changed the dangerous course of the rapid spread of the pandemic and reduced the number of people across the country The occurrence of 10,000 cases have won a valuable window for countries around the world to fight the pandemic. Finally, to provide support for the world's fight against the pandemic, China's manufacturing industry can significantly improve its ability to produce medical supplies in a relatively short period of time, and can meet the explosive demand caused by the pandemic. With the gradual improvement of the domestic pandemic, China has taken the initiative to assist other countries that need to protect materials. China is encouraging manufacturers of protective equipment, medical equipment, and therapeutic drugs to meet overseas demand and contribute to the global fight against this pandemic.

## Figures and Tables

**Figure 1:** The optimization path of China's international image.

**Figure 2:** SEIR model.

**Figure 3:** LS-Net overall framework.

**Figure 4:** Coronavirus disease (This picture is borrowed from the Internet).

**Figure 5:** Analysis of China's international image before and after the pandemic.

**Figure 6:** Comparison of the number of new cases per day in China and outside China.

**Figure 7:** The world's economy map (This picture is quoted from the Internet).

**Table 1:** Representative views of foreign scholars on the definition of national image.

years	Scholar	View
2003	Ale R. Holsti	It is believed that the international image is connected with the belief system of the country, and the international image is the “part of the belief system” formed by perceiving a country.
2010	Alpo Rusi	The international image is the image displayed by a sovereign country on the world stage and its reflection in international public opinion.
2012	Robert Jervis	The international image is defined as the image of a sovereign country in the flow of international news or in international news or speech reports.
2015	Gordeyeva	The international image is defined as the comprehensive evaluation and overall impression of other countries on the country, generally based on the international image reflected in the news media and public opinion of other countries.

**Table 2:** Differences in the mental health of the public in different regions under the pneumonia pandemic.

Subdimension	Outside Hubei province	Hubei province (not Wuhan)	Wuhan	*F*	*P*
	M (SD)	M (SD)	M (SD)		
Fear	2.67	2.56	2.79	1.15	0.54
Depression	1.89	1.99	2.34	3.43	0.05
Anxiety	3.14	3.23	3.18	0.13	0.87
Anger	3.21	2.99	3.16	1.69	0.21
*N*	811	666	654		

**Table 3:** Differences in the mental health of different genders in the pneumonia pandemic.

Area	Gender	Fear		Depression		Anxiety		Anger	
		*M*	SD	*M*	SD	*M*	SD	*M*	SD
Wuhan	Male	2.11	0.65	1.78	0.79	3.03	0.83	3.01	0.91
	Female	2.45	0.76	1.98	0.98	3.06	0.85	3.11	0.94
Hubei province (not Wuhan)	Male	2.65	0.87	1.87	0.91	3.01	0.89	3.02	0.90
	Female	2.42	0.88	1.96	0.75	3.11	0.87	3.06	0.93
Outside Hubei province	Male	2.52	0.89	1.89	0.76	3.12	0,91	3.03	0.95
	Female	2.34	0.91	1.99	0.78	3.08	0.87	3.08	0.92

**Table 4:** Differences in the mental health of different occupations under the pneumonia pandemic.

Sub-dimension	Student group	Staff member	*t*	*p*
	M (SD)	M (SD)		
Fear	2.54	2.13	0.78	0.44
Depression	1.78	1.78	−0.23	0.83
Anxiety	3.10	3.12	−1.41	0.11
Anger	3.03	3.10	−1.42	0.12
*N*	1881	231		

**Table 5:** Analysis of differences in mental health among people of different ages in the pandemic of pneumonia.

Subdimension	Under 20	20–29 years old	30–39 years old	Over 40 years old	F	*p*
	M (SD)	M (SD)	M (SD)	M (SD)		
Fear	2.33	2.61	2.13	2.23	2.00	0.12
Depression	1.91	1.91	1.89	1.87	0.21	0.78
Anxiety	3.10	3.11	3.11	3.11	2.11	0.10
Anger	3.01	3.09	3.10	2.78	1.11	0.32
*N*	1170	760	43	131		

## Data Availability

The data used to support the findings of this study can be obtained from the corresponding author upon request.
